This article has been retracted.

# MicroRNA-15b shuttled by bone marrow mesenchymal stem cell-derived extracellular vesicles binds to WWP1 and promotes osteogenic differentiation

**DOI:** 10.1186/s13075-020-02316-7

**Published:** 2020-11-16

**Authors:** Yanhong Li, Jing Wang, Yanchao Ma, Wenjia Du, Haijun Feng, Kai Feng, Guangjie Li, Shuanke Wang

**Affiliations:** Department of Orthopaedics, Lanzhou University Second Hospital, No. 82, Cuiyingmen, Chengguan District, Lanzhou, 730030 Gansu Province People’s Republic of China

**Keywords:** Osteogenic differentiation, Bone marrow mesenchymal stem cell, Extracellular vesicles, microRNA-15b, KLF2, WWP1, NF-κB signaling pathway

## Abstract

**Background:**

Osteogenic differentiation is an essential process for bone regeneration involving bone marrow mesenchymal stem cells (BMSCs). BMSC-secreted extracellular vesicles (EVs) enriched with microRNAs (miRs) have vital roles to play in mediating osteogenic differentiation. Therefore, this study aimed to explore the effect of BMSC-derived EVs loaded with miR-15b on osteogenic differentiation.

**Methods:**

Human BMSCs (hBMSCs) were cultured and treated with plasmids overexpressing or knocking down KLF2, WWP1, and miR-15b to define the role of derived EVs in osteogenic differentiation in vitro. The expression of osteogenic differentiation-related marker was measured by Western blot analysis. The interaction among miR-15b, WWP1, and ubiquitination of KLF2 was investigated by dual-luciferase reporter, immunoprecipitation, and GST pull-down assays. Moreover, EVs from hBMSCs transfected with miR-15b inhibitor (EV-miR-15b inhibitor) were injected into ovariectomized rats to verify the effect of miR-15b on bone loss in vivo.

**Results:**

WWP1 was downregulated, and KLF2 was upregulated during osteogenic differentiation. After co-culture with EVs, miR-15b expression was elevated and WWP1 expression was reduced in hBMSCs. Upregulation of miR-15b or KLF2 or downregulation of WWP1 or NF-κB increased ALP activity and cell mineralization, as well as osteogenic differentiation-related marker expression in hBMSCs. Mechanistically, miR-15b targeted and inhibited WWP1, thus attenuating KLF2 degradation and inhibiting NF-κB activity. Co-culture of EVs increased the bone volume and trabecular number, but decreased bone loss in ovariectomized rats, which could be reversed after treatment with EV-miR-15b inhibitor.

**Conclusion:**

Collectively, BMSC-derived EVs loaded with miR-15b promoted osteogenic differentiation by impairing WWP1-mediated KLF2 ubiquitination and inactivating the NF-κB signaling pathway.

**Graphical abstract:**

## Background

Osteoblasts and osteoclasts are responsible for bone turnover by mediating bone formation and bone resorption, respectively. Osteoblasts are derived from the osteogenic differentiation of mesenchymal stem cells (MSCs) in different regulatory processes [1]. Moreover, osteogenic differentiation of MSCs is a complex process, correlating to numerous environmental factors, like hormones and growth factors [2]. MSC osteogenic differentiation is pivotal for bone disease treatment and the repair of bone defect [3]. Furthermore, a prior study has documented the critical effects of human bone marrow MSC (hBMSC) osteogenic differentiation on bone regenerative therapies and regenerative potential of hBMSC-secreted extracellular vesicles (EVs) [4]. More importantly, it has been reported that BMSC-derived EVs could restore the BMSC function to suppress radiation-induced bone loss in rat models [5].

EVs are essential regulators and a critical means of intercellular communication, which are carriers of membrane cells and cytoplasmic proteins, lipids, and RNA [6]. It has been acknowledged that EVs secreted from various cells including BMSCs and osteoclasts, as well as the delivery of microRNAs (miRs) to osteoblasts, could regulate bone formation [7]. A study showed that miR-15b was observed in human MSC (hMSC)-secreted EVs [8]. The miR-15b is a member of the miR-15/107 group of miR genes that play an essential role in cell angiogenesis, stress response, metabolism, and division of vertebrate species [9]. Overexpression of miR-15b has been found during osteogenic differentiation of BMSCs in a previous study [10]. In our study, Starbase predicted the binding sites of miR-15b on the WW domain-containing E3 ubiquitin protein ligase 1 (WWP1) 3′-untranslated region (UTR). WWP1 encompasses an N-terminal C2 domain, four tandem WW domains for substrate binding, and a C-terminal catalytic HECT domain for ubiquitin transferring, which can function as the E3 ligase for PY motif-containing proteins, including Kruppel-like factor 5 (KLF5), and for non-PY motif-containing proteins-like KLF2 [11]. A prior study has identified the correlation between WWP1 and osteogenic differentiation of MSCs [12]. Meanwhile, it has been clarified that KLF2 could promote osteogenic differentiation in osteoblasts [13]. Moreover, WWP1 mediates both poly-ubiquitination and proteasomal degradation of KLF2 [14]. In this regard, we hypothesized that BMSC-secreted EVs mediated delivery of miR-15b might be involved in the osteogenic differentiation of BMSCs via the WWP1/KLF2 axis. In order to verify this hypothesis, we therefore provide functional evidence by performing overexpression and inhibition/silencing treatment, as well as co-culture in human bone marrow mesenchymal stem cells (hBMSCs) after osteogenic induction.

## Materials and methods

### Ethics approval

The animal experiments were approved by the Experimental Animal Ethics Committee of Lanzhou University Second Hospital (No. 2019A-224) and conducted in accordance with the *Guide for the Care and Use of Laboratory Animals* published by the National Institutes of Health. All efforts were made to minimize unnecessary distress to the animals.

### Culture of human bone marrow mesenchymal stem cells

The hBMSCs (ScienCell Research Laboratories, Carlsbad, CA, USA) were cultured in a 37 °C incubator with 5% CO_2_ with full relative humidity. For in vitro experiments, hBMSC incubation was performed with proliferation medium (PM) encompassing minimum essential medium α (α-MEM, Gibco, Carlsbad, CA, USA), 10% (v/v) fetal bovine serum (FBS, ScienCell Research Laboratories), and 100 IU/mL antibiotics (Gibco).

As for osteogenic induction, hBMSC culture was conducted with osteogenic medium (OM) encompassing standard PM, 10 mmol/L β-glycerophosphate, 0.2 mmol/L ascorbic acid, and 100 nmol/L dexamethasone. All other materials were bought from Sigma-Aldrich (St Louis, MO, USA) unless stated otherwise.

### Cell transfection

Small interfering RNA (siRNA) targeting WWP1 and negative control (NC) of siRNA (both from Santa Cruz Biotechnology Inc., Santa Cruz, CA, USA) were transfected into BMSCs under the mediation of DharmaFECT one transfection reagent (Thermo Scientific, Lafayette, CO, USA, www.dharmacon.com).

Based on the manuals provided by Lipofectamine 2000 (Invitrogen, Carlsbad, CA, USA), lentiviral vectors carrying short hairpin RNA (sh)-NC, sh-KLF2, overexpression (oe)-NC, oe-KLF2, and oe-WWP1 (Ribobio, Guangzhou, Guangdong, China) were transduced into BMSCs. Following 6 h, the medium was renewed, and cell culture was further conducted for 48 h.

Mimic-NC (100 nM), miR-15b mimic (100 nM), inhibitor-NC (100 nM) and, miR-15b inhibitor (100 nM) (Shanghai GenePharma Co., Ltd., Shanghai, China) were transfected into BMSCs by using Lipofectamine 2000 (Invitrogen). After 48 h of transfection, reverse transcription quantitative polymerase chain reaction (RT-qPCR) was performed to assess the transfection efficiency.

### Extraction of EVs from hBMSCs

FBS was centrifuged for 18 h at 100,000×*g* in advance to remove EVs from the serum to obtain an EV-free medium. The hBMSCs at 80% confluency were cultured in the EV-free medium for 48 h, followed by the collection of the supernatants. EVs were isolated from supernatants of hBMSCs through differential centrifugation and filtration steps. Specifically, cell supernatants were centrifuged at 2000×*g* for 20 min, then at 10,000×*g* for 40 min, followed by filtration using a 0.22-μm sterilized filter (Millipore, Bedford, MA, USA). After a 70-min ultracentifugation at 100,000×*g*, the supernatant was resuspended in phosphate-buffered saline (PBS) and centrifuged at 100,000×g for 70 min. After that, EVs were lysed in RIPA lysis buffer, followed by estimation of EV concentration based on the protocols of bicinchoninic acid (BCA) protein assay kit (Thermo Fisher Scientific Inc., Waltham, MA, USA).

### Identification of EVs from hBMSCs

A transmission electron microscopy (TEM) was adopted to measure the morphology of EVs. In brief, the hBMSC-derived EVs were fixed in 2% paraformaldehyde for 30 min and assembled on carbon-coated copper grids, followed by air-drying. The 1% uranyl acetate was employed twice for negative staining of the mixture. An HT7700 TEM (Hitachi High-Technologies Corporation, Tokyo, Japan) was adopted to capture images at 120 kV.

Nanoparticle tracking analysis (NTA) was applied for the evaluation of particle size and concentration of EVs. The ZetaView system (Particle Metrix GmbH, Microtrac, Meerbusch, Germany) was employed for the evaluation of EVs, followed by the result analysis by NTA analytical software (ZetaView, version 8.04.02). Western blot analysis was conducted to assess the protein expression of the specific markers (CD81, CD63), negative protein Calnexin, and co-expression protein tumor susceptibility gene 101 (TSG101) to identify EVs.

### Labeling and tracking of EVs from hBMSCs

hBMSCs and EVs were labeled based on the manuals of 3,3′-dioctadecyloxacarbocyanine perchlorate (CM-Dio) and 1,1′-dioctadecyl-3,3,3, 3′-tetramethylindocarbocyanine perchlorate (CM-DiI) (Beyotime Biotechnology, Haimen, China), respectively, followed by a 30-min culture in the dark at 37 °C. The unbound dye was removed by 70-min centrifugation at 100,000×*g* and 4 °C and 5-min centrifugation at 800×*g* at room temperature. Finally, EVs and BMSCs were mixed together, followed by a 24-h culture at 37 °C. The internalization of EVs was observed under fluorescence microscopy (Leica, Weltzlar, Germany), and images were analyzed using a Leica Application Suite Advanced Fluorescence (LASAF) software.

### Alkaline phosphatase activity measurement

Cells were cultured in OM for 7 days, followed by alkaline phosphatase (ALP) staining and quantitative analysis. The NBT/BCIP staining kit (Beijing Cowin Biotech Co., Ltd., Beijing, China) was utilized for ALP staining after cell fixation. According to the manufacturer’s instructions of the ALP active colorimetric quantitative detection kit (Nanjing Jiancheng Reagent Company, Nanjing, China), cells were centrifuged at 1000 rpm for 10 min and treated with Triton-X100. The optical density (OD) values were evaluated at 520 nm.

### Alizarin red S staining

hBMSCs were seeded onto six-well plates (1 × 10^5^ cells/well). Upon cell confluence, the medium was renewed to induction medium supplemented with 10 mmol/L β-glycerophosphate, 0.2 mmol/L ascorbic acid, and 100 nmol/L dexamethasone. The cells cultured for 14 days were subjected to Alizarin red S (ARS) staining as per the manufacturer’s instructions. In brief, the cells were washed three times with PBS, fixed using 4% paraformaldehyde (15 min), and stained with 0.2% ARS solution for 30 min. After washing three times with distilled water, the stained cells were photographed.

### RNA isolation and quantification

The RT-qPCR was initially carried out to determine the expression pattern of miR-15b in BMSCs at 7 days and 14 days of osteogenic differentiation. As per the manufacturer’s instructions, the TaqMan microRNA reverse transcription kit (Life Technologies, Carlsbad, CA, USA) was adopted to reversely transcribe small RNA samples (10 ng) into single-stranded cDNA. Real-time PCR amplification of miR was performed using TaqMan 2X universal PCR master mix and Applied Biosystems 7500 Fast Real-time PCR system (Applied Biosystems., Carlsbad, CA, USA). Each sample was subjected to three repeated RT-qPCR.

The RNeasy Mini Kit (Qiagen, Germantown, MD, USA, www.qiagen.com) was adopted for the isolation of total RNA. cDNA was synthesized using a MiRcute miRNA First-strand cDNA synthesis kit (Tiangen Biotech, Beijing, China) or Primer-Script TM one-step RT-qPCR kit (Takara, Shiga, Japan). Targets were amplified on an ABI7500 Real-Time PCR system (Applied Biosystems) using the SYBR Green I real-time PCR kit (Beijing Cowin Biotech Co., Ltd.). The relative expression level of mRNA or miR was normalized by glyceraldehyde-3-phosphate dehydrogenase (GAPDH) or U6 expression as internal controls. These values were then raised to the power of 2 (2^−ΔΔCt^) to yield fold expression relative to the reference point. The primers used are listed in Supplementary Table 1.

### Western blot analysis

Whole-cell lysates were prepared from the BMSCs. Cells were lysed using mammalian protein extraction reagent (Pierce Chemical, Dallas, TX), containing protease inhibitor mixture (Roche Applied Science, Indianapolis, IN). The whole-cell lysates (10 μg protein/lane) were loaded and separated in 10% sodium dodecyl sulfate-polyacrylamide gel electropheresis (SDS-PAGE) gels, electro-blotted into a nitrocellulose membrane, and immune-blotted with anti-rabbit antibodies (Abcam, Cambridge, UK) to GAPDH (ab181602, 1:10,000), KLF2 (ab139699, 1:1000), runt-related transcription factor 2 (Runx2, ab23981, 1:1000), osteocalcin (OCN, ab93876, 1:500), osteopontin (OPN, ab75285, 1:1000), WWP1 (ab43791, 1:1000), CD63 (ab134045, 1:1000), CD81 (ab109201, 1:1000), Calnexin (ab92573, 1:20,000), TSG101 (ab125011, 1:1000), p65 (ab32536, 1:1000), phosphorylated p65 (ab86299, 1:2000), IκBα (ab32518, 1:1000), and phosphorylated IκBα (ab133462, 1:10,000). The electrogenerated chemiluminescence (Amersham Biosciences, Piscataway, NJ, USA) was employed to visualize these bands.

### Dual-luciferase reporter assay

The Starbase software was utilized to predict the binding site between miR-15b and WWP1. The WWP1 3′-untranslated region (UTR) containing the predicted miR-15b binding sites was synthesized and subsequently cloned into a modified pcDNA3.1 plasmid containing a firefly luciferase reporter gene to construct a WWP1 wild-type (WT) luciferase reporter plasmid. The miR-375 binding site in the 3′-UTR of WWP1 was mutated with a site-directed mutagenesis kit (SBS Genetech Co., Ltd., Beijing, China), namely WWP1-mutant (MUT) luciferase reporter plasmid. All constructs were verified by DNA sequencing. The 293T cells were cultured in a 48-well plate when cells reached 70–80% confluence. Cells were co-transfected with 400 ng plasmids expressing WWP1-MUT or WWP1-WT and 40 ng firefly luciferase reporter plasmids or 4 ng pRL-TK, a plasmid-expressing Renilla luciferase (Promega, Madison, WI, USA). Following 24 h of transfection, the luciferase activity was detected on a Dual-Luciferase Reporter Assay System with values normalized to Renilla luciferase and depicted as fold change relative to basal activity.

The transcription activity of NF-κB was detected by using NF-κB luciferase reporter plasmid (YT451-BSJ, Beijing Biolab Technology Co., Ltd., Beijing, China).

### Immunoprecipitation and Western blot analysis

Anti-FLAG monoclonal antibody (F1804, Sigma-Aldrich), anti-Myc monoclonal antibody (m5546, Sigma-Aldrich), and immunoglobulin G (IgG) goat anti-rabbit polyclonal antibody (ab20272, 1:5000, Abcam) were applied to perform co-immunoprecipitation according to the standard protocol. Briefly, each 100-mm culture dish was cultured with 0.6 mL of 1× ice-cold cell lysis buffer containing 20 mM Tris-Cl (pH 7.5), 150 mM NaCl, 1 mM ethylene diamine tetraacetic acid (EDTA), 1 mM ethyleneglycol-bis (beta-aminoethylether)-*N*,*N*′-tetraacetic acid, 1% Triton X-100, 2.5 mM sodium pyrophosphate, 1 mM Na3VO4, 1 μg/mL leupeptin, and 1 mM fresh phenylmethylsulfonyl fluoride on ice for 5 min to the transfected BMSCs, and BMSCs in the plate were transferred to the fresh microcentrifuge tubes. Cell lysates were then sonicated 4 times (5 s each time) on ice and centrifuged for 10 min at 4 °C. The primary anti-Myc antibody (2 μL) was supplemented to 200 μL of culture supernatant overnight at 4 °C. The supernatant was then added with 30 μL of 50% protein A-agarose beads (Upstate, Waltham, MA, USA), followed by 2 h culture at 4 °C. Beads were washed with 500 μL of 1× cell lysis buffer for 5 times. Proteins were then resuspended in 50 μL of SDS sample buffer and analyzed by Western blot analysis.

### Glutathione-*S*-transferase pull-down assay

Glutathione-*S*-transferase (GST) fusion protein was purified from bacterial DNA fragments. After amplification, WWP1 was cloned into the pGEX-6p-1 GST fusion protein expression vector (Amersham Biosciences) and transformed into *Escherichia coli* strain BL21 (DE3, Stratagene, La Jolla, CA, USA). GST fusion protein was induced by 1 mM isopropyl-1-thio-β-d-galactopyranoside for 3 h at room temperature, followed by purification with 1 L glutathione-Sepharose 4B (Amersham Biosciences). The purified GST fusion protein was eluted into 10 mM reduced glutathione. The 10% SDS-PAGE and Coomassie Blue staining were conducted to identify the purity of the protein. With bovine serum albumin (Bio-Rad, Hercules, CA, USA) as a standard, the protein concentration was determined by the Bradford method. RNA transcription and protein translation were carried out in vitro using [35S] methionine (Amersham Biosciences) following the manufacturer’s instructions of TNT Quick-coupled Transcription/Translation systems (Promega).

Equal molar amounts of purified GST fusion proteins (GST, GST-WWP1) were fixed using 0.5 mL GST pull-down binding buffer containing 10 mM 4-(2-hydroxyethyl)-1-piperazineëthanesulfonic acid (pH 7.6), 3 mM MgCl2, 100 mM KCl, 5 mM EDTA, 5% glycerol, and 0.5% CA630, and the solution was added into 50 μL of 50% glutathione-Sepharose 4B suspended beads (Amersham Biosciences). Following 1 h of culture at 4 °C with rotation, beads were washed 3 times with GST pull-down binding buffer and recovered with 0.5 mL GST pull-down binding buffer. The 10-μL 35 S-labeled in vitro-translated protein (KLF2) was supplemented and mixed for 2 h at 4 °C with rotation.

The beads were then washed twice with 0.5 mL ice-cold radioimmune precipitation assay buffer and 1 mL cold PBS, respectively. The bound proteins were eluted with 30 μL boiled loading buffer. Coomassie Blue staining was performed and the GST protein was observed, followed by autoradiography to measure the 35 S-labeled protein. The in vitro ubiquitination assay was carried out using the Ubiquitin-Protein Conjugation kit (BostonBiochem, Cambridge, MA, USA). Briefly, 2 μL of rabbit reticulocyte lysate-translated 35 S-labeled KLF2 was incubated in the absence or presence of GST-WWP1 (2.5 μg), 8 μg fraction A, 8 μg fraction B, 26 μg ubiquitin, 4 μM ubiquitin aldehyde, and 2.5 μL energy solution (10×) in a 25-μL system, followed by a 30-min culture at 37 °C. The reaction was terminated with the addition of 25 μL of 3× sample loading buffer. Samples were electrophoresed on 10% SDS-polyacrylamide gels and analyzed by autoradiography.

### In vivo ubiquitination analysis

The 293T cells were transfected with hemagglutinin (HA)-ubiquitin, Myc-WWP1, and either Flag-KLF2 or Flag-KLF2-MUT, followed by treatment with 10 μM MG132 for 4 h, and harvested. Cells were lysed in 100 μL of regular lysis buffer. The cell lysates were denatured at 95 °C for 5 min with the presence of 1% SDS, followed by overnight culture in anti-Flag antibody and protein G-agarose (Sigma-Aldrich, www.sigmaaldrich.com) overnight at 4 °C. Western blot analysis with an anti-HA antibody was conducted to analyze the immunoprecipitates.

BMSCs were first treated with 10 μM MG132 (MedChemExpress, Shanghai, China) for 4 h. Cell lysates were then cultured with anti-KLF2 antibody and protein G agarose overnight at 4 °C. The endogenous ubiquitination of KLF2 in the immunoprecipitates was assessed by Western blot analysis with the use of an anti-ubiquitin antibody.

### Protein half-life assay

Cells were treated with 10 μM cycloheximide (CHX, MedChemExpress) for different times, or cells were treated with MG132 at the same time to prepare crude extracts. The protein levels were then determined by Western blot analysis.

### Establishment of ovariectomized rat model

All the operations on rats were carried out under general anesthesia and sterile conditions, and the postoperative analgesia nursing was performed using anti-amine phencycline. In this study, a total of 40 female Sprague-Dawley rats (Tengxin Biotechnology Co., Ltd., Chongqing, China) aged 3 months were selected, among which, 8 rats received sham operation and 32 rats were used for induction of ovariectomized (OVX) models. In brief, rats were anesthetized by 30 mg/kg pentobarbital sodium, followed by the preparation of 10-mm bilateral lumbar lateral skin linear incision. After exposing the muscles and peritoneum by blunt dissection, bilateral ovaries were gently excised. All sham-operated rats underwent a similar procedure, except for the removal of bilateral ovaries. After the tissues were repositioned and sutured into the synthetic layer, the rats were injected with 40,000 IU/mL penicillin at 1 mL/kg for 3 days. After OVX model establishment, OVX rats were injected with 20 μL of PBS, 20 μL of EVs suspension derived from BMSCs (BMSC-EVs), 20 μL of EVs suspension isolated from BMSCs transfected with inhibitor NC using liposomes (EV-inhibitor NC), or 20 μL of EVs suspension isolated from BMSCs transfected with miR-15b inhibitor using liposomes (EV-miR-15b inhibitor) through the periosteum of the bone marrow cavity of femur twice in a week [15] (8 rats for each injection). After 3 weeks, the distal femur was taken and subjected to micro-CT and HE staining to observe the tissue morphology [16, 17].

### Micro-CT analysis

Three weeks later, the micro-CT system (mCT-80, Scanco medical, Brüttisellen, Switzerland) was adopted to analyze the changes of the microstructure and the formation of new bone in the defected area. In the medium-resolution mode, the samples were scanned with a thickness of 0.018 mm per slice, a 1024-reconstruction matrix, and 200-ms integration time. After 3D reconstruction, bone mineral density (BMD), the ratio of bone volume to total tissue volume (BV/TV), trabecular number (Tb.N), trabecular thickness (Tb.Th), and connective density (Conn.D) were automatically determined.

### Statistical analysis

All measurement data were shown as mean ± standard deviation and analyzed by SPSS 19.0 software (IBM, Armonk, NY, USA), with a level of significance set at *p* < 0.05. Conforming to the normal distribution and homogeneity of variance, data between the two groups were compared by independent sample *t* test. Comparisons among multiple groups were performed using one-way analysis of variance (ANOVA), followed by Tukey’s post hoc test, and data comparison among the groups at different time points was analyzed by repeated-measures ANOVA, followed by Tukey’s post hoc test.

## Results

### miR-15b directly targets WWP1 3′-UTR

The expression of miR-15b in BMSCs with osteogenic differentiation for 0, 7, and 14 days was determined by the TaqMan probe, demonstrating that the expression of miR-15b increased significantly with the osteogenic differentiation of BMSCs in a time-dependent manner (Supplementary Figure 1). According to the Starbase prediction software, miR-15b directly targeted WWP1 3′-UTR (Fig. 1a). A dual-luciferase reporter assay was conducted to verify the targeting relationship, and the results showed that in HEK-293T cells, miR-15b mimic diminished the luciferase activity of WWP1 3′-UTR (WT) (Fig. 1b). Besides, RT-qPCR results revealed that increased expression of miR-15b and the decreased expression of WWP1 were observed in BMSCs after miR-15b mimic transfection (Fig. 1c). Meanwhile, Western blot analysis demonstrated that WWP1 was downregulated in miR-15b mimic-transfected BMSCs (Fig. 1d). Therefore, these results suggested that miR-15b could target and negatively regulate WWP1.

**Fig. 1:** WWP1 is targeted and negatively regulated by miR-15b. **a** The binding of miR-15b to WWP1 3′-UTR predicted by Starbase software. **b** The targeting relationship between miR-15b and WWP1 evaluated by dual-luciferase reporter assay. **c** miR-15b expression and WWP1 mRNA expression in BMSCs after transfection with mimic-NC or miR-15b mimic detected by RT-qPCR normalized to U6 and GAPDH. **d** WWP1 protein expression in BMSCs after transfection with mimic-NC or miR-15b mimic detected by Western blot analysis normalized to GAPDH. The measurement data were shown as mean ± standard deviation and compared by independent sample *t* test. The cell experiment was repeated three times. *p < 0.05 vs. transfection with mimic-NC

### BMSC-derived EVs loaded with miR-15b suppress WWP1 expression in BMSCs

Next, we moved to explore the effects of BMSC-derived EVs loaded with miR-15b on WWP1 expression. EVs were first isolated from BMSCs by high-speed centrifugation, and the structure was round or oval with a double-layer membrane (Fig. 2a). NTA analysis documented that the size of the EVs was mainly about 100 nm (Fig. 2b). Western blot analysis of the isolated EVs demonstrated that CD63 and CD81 only existed in the EVs, whereas Calnexin was expressed only in the lysate, and TSG101 was expressed in both EVs and lysate (Fig. 2c). After BMSCs were cultured with the isolated EVs, RT-qPCR displayed that miR-15b expression was significantly enhanced (Fig. 2d). In order to determine the uptake of EVs by BMSCs, BMSCs and EVs were labeled with fluorescent carbocyanine dyes CM-Dio (green) and CM-Dil (red), respectively. After 24 h of co-culture, the distribution of EVs in BMSCs was observed by a fluorescence microscope. The results depicted that the EVs were successfully absorbed by BMSCs (Fig. 2e). EVs were then extracted from BMSCs and transfected with inhibitor-NC or miR-15b inhibitor (EV-inhibitor-NC or EV-miR-15b inhibitor), followed by supplementation into hBMSCs. The results demonstrated that the co-culture of EVs elevated miR-15b expression but diminished WWP1 expression in BMSCs, which was opposite after the treatment with EV-miR-15b inhibitor (Fig. 2f, g). Taken together, these results suggested that WWP1 expression in BMSCs could be reduced by BMSC-derived EVs loaded with miR-15b.

**Fig. 2:** BMSC-secreted EVs mediated delivery of miR-15b reduces WWP1 expression in BMSCs. **a** The structure of EVs observed under a TEM (scale bar = 100 nm). **b** The size of EVs detected by NTA. **c** The expression of CD63, CD81, Calnexin, and TSG101 in EVs and lysate detected by Western blot analysis normalized to GAPDH. **d** miR-15b expression in BMSCs after co-culture with BMSC-derived EVs determined by RT-qPCR normalized to U6. *p < 0.05 vs. hBMSCs. **e** The uptake of EVs by BMSCs observed under a fluorescence microscope (× 400). **f** miR-15b expression in BMSCs after co-culture with inhibitor-NC, EV-inhibitor-NC, or EV-miR-15b inhibitor determined by RT-qPCR normalized to U6. **g** WWP1 expression in BMSCs after co-culture with inhibitor-NC, EV-inhibitor-NC, or EV-miR-15b inhibitor determined by Western blot analysis normalized to GAPDH. *p < 0.05 vs. hBMSCs treated with inhibitor NC. ^#^*p* < 0.05 vs. hBMSCs treated with EV-inhibitor-NC. The measurement data were shown as mean ± standard deviation. Data between the two groups were compared by independent sample *t* test. Comparisons among multiple groups were performed using one-way ANOVA, followed by Tukey’s post hoc test. The cell experiment was repeated three times

### KLF2 is ubiquitinated and degraded by E3 ubiquitin ligase WWP1 in BMSCs

A prior study has identified that the correlation between WWP1 and osteogenic differentiation of MSCs [12]. Moreover, WWP1 mediates both poly-ubiquitination and proteasomal degradation of KLF2 [14]. In order to determine the endogenous target of WWP1 in BMSCs, the protein level of KLF2 was detected. In cells treated with CHX, the protein level of KLF2 was diminished as time went on, while the decrease of KLF2 protein level was decelerated with the prolongation of time in cells with CHX-MG132 (Fig. 3a). After overexpression of ubiquitin ligases Smurf1, Smurf2, Itch, and WWP1, the protein level of KLF2 decreased only in cells overexpressing WWP1 (Fig. 3b), while in the cells with MG132, the decrease of KLF2 protein level was inhibited (Fig. 3c). IP and GST pull-down assays were performed with the presence of proteasome inhibitor MG132 to detect the interaction between WWP1 and KLF2 at the protein level. Myc-labeled WWP1 was expressed in the cells, and endogenous KLF2 was detected. As shown in Fig. 3d, Myc-WWP1 was immunoprecipitated by the anti-KLF2 antibody, but not by IgG control. These results indicated that WWP1 interacted with endogenous KLF2 in BMSCs. As documented in Fig. 3e, GST-WWP1 fusion protein and KLF2 protein translated in vitro were used for the GST pull-down experiment. The results demonstrated that WT GST-WWP1 pulled down KLF2 protein, but under the same conditions, the single GST protein did not bind to KLF2 protein. Under the condition of IP experiment with FLAG, a ubiquitination experiment was carried out and ubiquitin UB was added to detect the ubiquitination of KLF2 after overexpression of WWP1, as depicted in Fig. 3f. WWP1 was used to induce the ubiquitination of endogenous KLF2 protein. After treatment with MG132 (10 μM, 4 h), Western blot analysis was conducted with the use of an anti-KLF2 antibody. After treatment with Myc-labeled WWP1, the ubiquitination and degradation of KLF2 by WWP1 was detected. These results suggested that KLF2 could be ubiquitized and degraded by E3 ubiquitin ligase WWP1.

**Fig. 3:** E3 ubiquitin ligase WWP1 promotes ubiquitination and degradation of KLF2 in BMSCs. **a** The protein level of KLF2 in BMSCs after treatment with CHX or CHX-MG132. *p < 0.05 vs. DMSO. ^#^*p* < 0.05 vs. CHX. **b** The protein level of KLF2 after overexpression of ubiquitin ligases Smurf1, Smurf2, Itch, and WWP1 measured by Western blot analysis normalized to GAPDH. *p < 0.05 vs. oe-NC. **c** The protein level of KLF2 after overexpression of WWP1 and treatment with MG132 measured by Western blot analysis normalized to GAPDH. **d** The effects of Myc-labeled WWP1 on endogenous KLF2. The input was the positive control, and IgG was the negative control. **e** Exogenous KLF2 assessed by GST pull-down assay with GST-WWP1 fusion protein and KLF2 protein translated in vitro. The input was the positive control, and GST was the negative control. **f** Ubiquitination of KLF2 by adding ubiquitin UB after overexpression of WWP1. *p < 0.05 vs. oe-NC + DMSO. ^#^*p* < 0.05 vs. oe-WWP1 + DMSO. **g** WWP1 protein level during osteogenic differentiation measured by Western blot analysis normalized to GAPDH. *p < 0.05 vs. PM. **h** Silencing efficiency of WWP1 evaluated by Western blot analysis normalized to GAPDH. **i**, **j** ALP activity of si-WWP1-transfected BMSCs (× 200). **k** The expression of osteogenic differentiation-related marker proteins (Runx2, OPN, and OCN) in si-WWP1-transfected BMSCs with osteogenic differentiation for 14 days evaluated by Western blot analysis normalized to GAPDH. *p < 0.05 vs. sh-NC. ^#^*p* < 0.05 vs. hBMSCs treated with EV-inhibitor-NC. **l** The mineralization of BMSCs determined using ARS staining after treatment with si-WWP1 or si-NC. *p < 0.05 vs. BMSCs transfected with si-NC (× 200). The measurement data were shown as mean ± standard deviation. Data between the two groups were compared by independent sample *t* test. Comparisons among multiple groups were performed using one-way ANOVA, followed by Tukey’s post hoc test. Data comparison among the groups at different time points was analyzed by repeated-measures ANOVA, followed by Tukey’s post hoc test. The cell experiment was repeated three times

In addition, Western blot analysis detected that the protein level of WWP1 was diminished during osteogenic differentiation (Fig. 3g). Subsequently, the stably transfected BMSCs with si-WWP1 was constructed and was confirmed by Western blot analysis (Fig. 3h). The transfected cells were induced to differentiate into osteoblasts. The results of ALP showed that the ALP staining and the activity of si-WWP1-transfected BMSCs were increased significantly (Fig. 3i, j). Western blot analysis displayed that the expression of marker proteins (Runx2, OPN, and OCN) of BMSC osteogenic differentiation in si-WWP1-transfected BMSCs enhanced significantly (Fig. 3k). Further, the ARS staining exhibited that si-WWP1 treatment increased the mineralization of BMSCs, as compared with si-NC (Fig. 3l). Hence, these results suggested that E3 ubiquitin ligase WWP1 could ubiquitize and degrade KLF2 in BMSCs.

### KLF2 promotes osteogenic differentiation by inhibiting the transcription activity of NF-κB in BMSCs

Western blot analysis was performed to detect the protein expression of KLF2 in the process of osteoblasts differentiation. As described in Fig. 4a, KLF2 expression was significantly enhanced during osteogenic differentiation. BMSCs were treated with oe-KLF2, sh-KLF2-1 or sh-KLF2-2, and sh-KLF2-1 with high transfection efficiency was selected as sh-KLF2 for subsequent experiments (Fig. 4b). Western blot analysis was performed to detect the transfection efficiency of KLF2. The results revealed that KLF2 expression was significantly reduced after sh-KLF2 treatment and elevated obviously after oe-KLF2 transduction. After the induction of osteogenic differentiation, the results of ALP staining indicated that the ALP staining and the activity of BMSCs were notably decreased by the silencing of KLF2 but was remarkably increased by overexpressing KLF2 (Fig. 4c, d). Then, Western blot analysis displayed that KLF2 silencing was significantly reduced, but KLF2 overexpression resulted in enhanced expression of Runx2, OPN, and OCN in BMSCs (Fig. 4e). ARS staining displayed that sh-KLF2 treatment reduced the mineralization of BMSCs, whereas oe-KLF2 elevated the mineralization of BMSCs (Fig. 4f). Since the NF-κB signaling pathway involved the activation of NF-κB, p65 was used as an activator of NF-κB to conduct dual-luciferase reporter assay. The results showed that the luciferase activity was remarkably diminished by treatment with p65, which was abrogated by overexpressing KLF2 (Fig. 4g), indicating that KLF2 could inactivate the NF-κB signaling pathway through p65. Subsequently, Tanshinone-I (NF-κB inhibitor) was added to the BMSCs with KLF2 silencing. Tanshinone-I promoted ALP activity, and the expression of Runx2, OPN, and OCN in BMSCs with KLF2 silencing was observed. Meanwhile, TNF-α, a NF-κB activator, was added to the BMSCs overexpressing KLF2. In BMSCs overexpressing KLF2, ALP activity and the expression of Runx2, OPN, and OCN were significantly diminished upon TNF-α treatment (Fig. 4h–j). ARS staining displayed that co-treatment of sh-KLF2 and Tanshinone-I increased the mineralization of BMSCs compared with sh-KLF2 alone, whereas mineralization of BMSCs was reduced in response to co-treatment of oe-KLF2 and TNF-α, as compared with oe-KLF2 alone (Fig. 4k). The abovementioned results suggested that KLF2 could repress the transcription activity of NF-κB to induce osteogenic differentiation in BMSCs.

**Fig. 4:** KLF2 overexpression promotes osteogenic differentiation in BMSCs by suppressing the transcription activity of NF-κB. **a** The protein expression of KLF2 during osteoblasts differentiation assessed by Western blot analysis normalized to GAPDH. *p < 0.05 vs. PM. **b** KLF2 expression in BMSCs after transduction with oe-KLF2, sh-KLF2-1, or sh-KLF2-2. **c**, **d** ALP activity in BMSCs after the alteration of KLF2 (× 200). **e** The expression of Runx2, OPN, and OCN in BMSCs with osteogenic differentiation for 14 days after the alteration of KLF2 assessed by Western blot analysis normalized to GAPDH. *p < 0.05 vs. BMSCs transfected with sh-NC. ^#^*p* < 0.05 vs. BMSCs transfected with oe-NC. **f** The mineralization of BMSCs determined using ARS staining after treatment with sh-NC, sh-KLF2, oe-NC, or oe-KLF2. *p < 0.05 vs. BMSCs treated with sh-NC. ^#^*p* < 0.05 BMSCs treated with oe-NC (× 200). **g** The interaction of KLF2 with NF-κB detected by dual-luciferase reporter assay. *p < 0.05 vs. oe-NC. ^#^*p* < 0.05 vs. p65 + oe-NC. **h**, **i** ALP activity in BMSCs after the alteration of KLF2 and NF-Κb (× 200). **j** The expression of Runx2, OPN, and OCN in BMSCs with osteogenic differentiation for 14 days after the alteration of KLF2 and NF-κB measured by Western blot analysis normalized to GAPDH. *p < 0.05 vs. BMSCs transduced with sh-KLF2. ^#^*p* < 0.05 vs. BMSCs transduced with oe-KLF2. **k** The mineralization of BMSCs determined using ARS staining after treatment with sh-KLF2 + Tanshinone-I, sh-KLF2, oe-KLF2 + TNF-α, or oe-KLF2 (× 200). *p < 0.05 vs. BMSCs transduced with sh-KLF2. ^#^*p* < 0.05 BMSCs transduced with oe-KLF2. The measurement data were shown as mean ± standard deviation. Data between the two groups were compared by independent sample *t* test. Comparisons among multiple groups were performed using one-way ANOVA, followed by Tukey’s post hoc test. The cell experiment was repeated three times

### NF-κB signaling pathway inhibits osteogenic differentiation of BMSCs

Tanshinone-I and TNF-α were used to explore the effect of the NF-κB signaling pathway on the osteogenic differentiation of BMSCs. Western blot analysis documented that TNF-α treatment resulted in diminished IκBα expression, unchanged p65 expression, and increased phosphorylation of IκBα and p65 in BMSCs, whereas Tanshinone-I did not affect the expression of IκBα and p65, but resulted in reduced phosphorylation of IκBα and p65 in BMSCs (Fig. 5a). Meanwhile, the levels of TNF-α were remarkably diminished, but Tanshinone-I resulted in enhanced ALP activity in BMSCs (Fig. 5b, c). Besides, Western blot analysis depicted that the expression of Runx2, OPN, and OCN in BMSCs was diminished by TNF-α but was elevated by Tanshinone-I (Fig. 5d). ARS staining demonstrated that TNF-α treatment reduced the mineralization of BMSCs compared with PBS treatment, while Tanshinone-I treatment augmented mineralization of BMSCs in comparison with DMSO (Fig. 5e). In summary, these results suggested that NF-κB signaling pathway activation could suppress the osteogenic differentiation of BMSCs.

**Fig. 5:** Activation of the NF-κB signaling pathway leads to the repression of osteogenic differentiation of BMSCs. BMSCs were treated with PBS, TNF-α, DMSO, or Tanshinone-I. **a** The expression of IκBα and p65, as well as phosphorylation of IκBα and p65 in BMSCs evaluated by Western blot analysis normalized to GAPDH. **b**, **c** ALP activity in BMSCs (× 200). **d** The expression of Runx2, OPN, and OCN in BMSCs with osteogenic differentiation for 14 days assessed by Western blot analysis normalized to GAPDH. *p < 0.05 vs. BMSCs treated with PBS. ^#^*p* < 0.05 vs. BMSCs treated with DMSO. **e** The mineralization of BMSCs determined using ARS staining after treatment with TNF-α, PBS, Tanshinone-I, or DMSO (× 200). *p < 0.05 vs. BMSCs treated with PBS. ^#^*p* < 0.05 BMSCs treated with DMSO. The measurement data were shown as mean ± standard deviation and compared by independent sample *t* test. The cell experiment was repeated three times

### BMSC-derived EVs loaded with miR-15b regulate the KLF2/NF-κB axis by targeting WWP1 to promote osteogenic differentiation of BMSCs

EVs were extracted from BMSCs transfected with inhibitor-NC or miR-15b inhibitor (EV-inhibitor-NC or EV-miR-15b inhibitor) and subsequently co-cultured with hBMSCs, followed by osteogenic differentiation induction. The transfection efficiency of miR-15b inhibitor was shown in Fig. 2f. Moreover, the co-culture of EVs resulted in strengthened ALP activity in BMSCs, where opposite results were observed in response to EV-miR-15b inhibitor (Fig. 6a, b). Western blot analysis demonstrated that WWP1 expression was significantly decreased but the expression of KLF2, Runx2, OPN, and OCN in BMSCs was remarkably enhanced by EVs, where opposite changes were observed after EV-miR-15b inhibitor treatment (Fig. 6c, d). ARS staining demonstrated that the co-culture of EVs enhanced the mineralization of BMSCs, while the treatment of hMSCs + EV + miR-15b inhibitor reduced the mineralization of BMSCs (Fig. 6e). According to the results from dual-luciferase reporter assay, NF-κB activity was significantly decreased in BMSCs in response to EVs, while NF-κB activity was notably elevated in EV-miR-15b inhibitor-treated BMSCs (Fig. 6f). These results demonstrated that BMSC-derived EVs loaded with miR-15b could promote osteogenic differentiation of BMSCs by regulating the KLF2/NF-κB axis via WWP1.

**Fig. 6:** BMSC-derived EVs loaded with miR-15b induce osteogenic differentiation of BMSCs by inactivating the KLF2-dependent NF-κB signaling pathway via targeting WWP1. BMSCs were co-cultured with inhibitor NC, EV-inhibitor NC, or EV-miR-15b inhibitor. **a**, **b** ALP activity in BMSCs (× 200). **c**, **d** The expression of WWP1, KLF2, Runx2, OPN, and OCN in BMSCs with osteogenic differentiation for 14 days assessed by Western blot analysis normalized to GAPDH. **e** The mineralization of BMSCs determined using ARS staining after treatment with hMSCs + inhibitor-NC, hMSCs + EV + inhibitor-NC, hMSCs + EV + inhibitor-NC, or hMSCs + EV + miR-15b inhibitor (× 200). *p < 0.05 vs. hMSCs + inhibitor-NC; ^#^*p* < 0.05 vs. hMSCs + EV + inhibitor-NC. **f** NF-κB activity in BMSCs evaluated by dual-luciferase reporter assay. *p < 0.05 vs. BMSCs treated with inhibitor NC. ^#^*p* < 0.05 vs. BMSCs treated with EV-inhibitor NC. The measurement data were shown as mean ± standard deviation and compared by one-way ANOVA, followed by Tukey’s post hoc test. The cell experiment was repeated three times

### BMSC-derived EVs loaded with miR-15b alleviate bone loss in OVX rats

OVX model was induced on rats to investigate the effect of BMSC-derived EVs loaded with miR-15b on osteogenic differentiation in vivo. After the establishment of the model for 2 months, the tibia was collected and subjected to micro-CT and histomorphological analysis. HE staining demonstrated that compared with sham-operated rats, the bone volume and the trabecular number of OVX rats were potently reduced, but the bone marrow fat was increased. The co-culture of EVs resulted in increased bone volume and trabecular number but decreased bone marrow fat in OVX rats, where opposite results were detected after treatment with EV-miR-15b inhibitor (Fig. 7a). Similar results were observed by CT 3D reconstruction (Fig. 7b). These results indicated that the BMSC-derived EVs could reduce bone loss in rats. To quantify these changes, analyze 12.0 software was adopted to analyze the bone microstructure. As described in Fig. 7c–g, on the 28th day, the levels of BMD, BV/TV, Tb.N, Tb.Th, and Conn.D were significantly lower in OVX rats than in sham-operated rats. However, BMD, BV/TV, Tb.N, Tb.Th, and Conn.D were remarkably enhanced by the treatment with EVs, while treatment upon EV-miR-15b inhibitor resulted in opposite results. Together, the abovementioned results indicated that BMSC-derived EVs loaded with miR-15b could reduce bone loss in OVX rats.

**Fig. 7:** Bone loss was suppressed by BMSC-derived EVs loaded with miR-15b in OVX rats. Sham-operated rats were used as controls, while OVX rats were treated with or without EVs, EV-inhibitor NC, or EV-miR-15b inhibitor. **a** The morphology of rat tibia observed by HE staining (× 200). **b** Micro-CT analysis of tibia tissues of rats. **c** BV/TV of rats. **d** BMD of rats. **e** Tb.N of rats. **f** Tb.Th of rats. **g** Conn.D of rats. *p < 0.05 vs. sham-operated rats. ^#^*p* < 0.05 vs. OVX rats. ^&^*p* < 0.05 vs. OVX rats treated with EV-inhibitor NC. The measurement data were shown as mean ± standard deviation and compared by one-way ANOVA, followed by Tukey’s post hoc test. *n* = 8

## Discussion

Osteogenic differentiation of BMSCs has been well documented to correlate to the formation and remodeling of the bone [18]. Moreover, postmenopausal osteoporosis can also be caused by the repression of BMSC osteogenic differentiation [19]. Therefore, the osteogenic differentiation of BMSCs may be a potential target in the treatment of bone disease. A previous study has revealed that BMSC-secreted EVs were elucidated to regulate the osteogenic differentiation of BMSCs [20]. Meanwhile, miRs also serve as modulators of osteogenic differentiation of BMSCs [21]. Therefore, this study was intended to explore the potential regulatory role of BMSC-derived EVs loaded with miR-15b in osteogenic differentiation. Together, the obtained findings revealed the promoting effects of BMSC-derived EVs loaded with miR-15b on osteogenic differentiation of BMSCs via the WWP1/KLF2/NF-κB axis.

The present study revealed that WWP1 was under-expressed, but KLF2 was highly expressed in osteodifferentiated BMSCs, whereas WWP1 promoted ubiquitination and degradation of KLF2 to activate the NF-κB signaling pathway, thereby suppressing osteogenic differentiation of BMSCs. As an E3 ubiquitin ligase, inhibition of WWP1 has been reported to promote osteoblast activity and matrix mineralization [22]. Another prior study revealed that WWP1 could repress osteoblast differentiation and migration to inversely modulate osteoblast function [23]. More importantly, Zhao et al. reported that WWP1 elevated ubiquitination and degradation of JunB which positively mediated osteoblast differentiation [12], indicating that WWP1 upregulation may contribute to the repression of osteogenic differentiation. Besides, our results were supported by a previous study whereby WWP1 promoted ubiquitination and degradation of KLF2 [14]. KLF2 has been revealed to play an important role in maintaining the stemness of hMSCs during bone regeneration [24]. Similarly, the silencing of KLF2 has been reported to repress osteoblast differentiation [25]. Furthermore, the upregulation of KLF2 has been detected in the osteogenic differentiation process in previous work done by Hou et al. [13]. The suppressive effects of KLF2 on the transcriptional activity of NF-κB in monocytes have also been reported in previous literature [26], which was in line with our results. In fact, several studies have shown the effect of the NF-κB signaling pathway on osteogenic differentiation. For instance, the osteogenic differentiation of pre-osteoblasts was repressed through the activation of the NF-κB signaling pathway [27]. Another study evidenced that the taxifolin-inactivated NF-κB signaling pathway promoted osteogenic differentiation of hBMSCs [28]. Therefore, it was suggested that osteogenic differentiation of hBMSCs could be regulated by the WWP1/KLF2/NF-κB axis.

Subsequently, it is well-known that miRs can bind to the complementary sequences in the 3′-UTR of their target mRNAs to inversely regulate gene expression, which triggers mRNA degradation or translation repression [29]. In a previous study, miR-15b has been shown to directly target 3′-UTR of SMAD3 to downregulate SMAD3 in nucleus pulposus cells [30]. Also, it has been reported that miR-452could directly target WWP1 in prostate cancer cells [31], which partially supported our results that miR-15b could target and negatively regulate WWP1 to promote osteogenic differentiation of hBMSCs. Similarly, another prior research unraveled that miR-15b overexpression resulted in osteogenic differentiation of hBMSCs by targeting SMAD7 to alleviate steroid-induced osteonecrosis of the femoral head [32]. Moreover, miR-15b overexpression has been reported to increase osteoblast differentiation by activating Runx2, an osteoblast differentiation-related marker gene [33]. In our study, BMSC-derived EVs loaded with miR-15b regulated the KLF2/NF-κB axis by targeting WWP1 to promote osteogenic differentiation of BMSCs in vitro and attenuated bone loss in vivo. Due to the available osteogenic potential and abundant source, BMSCs have been regarded as the most promising cell type in bone regeneration [34]. BMSC-secreted EVs also possess osteogenic effects to relieve steroid-induced femoral head necrosis [35]. BMSC-derived EVs could alleviate bone loss caused by radiation in rats through the restoration of the BMSC function [5]. Another recent research has suggested that miR-15b was present in hMSC-secreted EVs [8]. In addition, another research uncovered that BMSC-secreted EVs could increase the expression of ALP, OCN, OPN, and Runx2 to induce osteogenic differentiation of BMSCs via miR-196a [20]. Hence, BMSC-derived EVs loaded with miR-15b might promote osteogenic differentiation of BMSCs via the WWP1/KLF2/NF-κB axis.

## Conclusion

In summary, the present study provides evidence on the function of BMSC-derived EVs containing miR-15b on the osteogenic differentiation. BMSC-secreted EVs carrying miR-15b could target WWP1 to inhibit the ubiquitination and degradation of KLF2, thereby inactivating the NF-κB signaling pathway in BMSCs to induce osteogenic differentiation. Collectively, our results suggest that BMSC-derived EVs containing miR-15b may be a potential novel tool for therapeutic strategies to prevent bone loss. However, further in vivo and in vitro investigations are still required to elucidate the specific molecular mechanism of the miR-15b/WWP1/KLF2/NF-κB network underlying osteogenic differentiation and bone loss.

## Supplementary information

**Additional file 1: Supplementary Figure 1.** The expression of miR-15b in BMSCs after osteogenic differentiation at 0, 7 days and 14 days. The expression of miR-15b in BMSCs after osteogenic differentiation at 0, 7 days and 14 days determined using Taq-Man RT-qPCR. The experiment was repeated three times. * *p* < 0.05 vs. 0 day. The measurement data were shown as mean ± standard deviation and compared by one-way ANOVA, followed by Tukey’s post-hoc test.

**Additional file 2: Supplemental Table 1.** Primer sequences for RT-qPCR.

## Data Availability

The datasets generated/analyzed during the current study are available.

## Abbreviations

BMSCs: Bone marrow mesenchymal stem cells
miRs: MicroRNAs
EVs: Extracellular vesicles
MSCs: Mesenchymal stem cells
WWP1: WW domain-containing E3 ubiquitin protein ligase 1
UTR: Untranslated region
KLF5: Kruppel-like factor 5
hBMSCs: Human bone marrow mesenchymal stem cells
PM: Proliferation medium
OM: Osteogenic medium
siRNA: Small interfering RNA
NC: Negative control
Sh: Short hairpin RNA
Oe: Overexpression
PBS: Phosphate-buffered saline
TEM: Transmission electron microscopy
NTA: Nanoparticle tracking analysis
TSG101: Tumor susceptibility gene 101
LASAF: Leica Application Suite Advanced Fluorescence
ALP: Alkaline phosphatase
OD: Optical density
WT: Wild-type
MUT: Mutant
EDTA: Ethylene diamine tetraacetic acid
GST: Glutathione-*S*-transferase
HA: Hemagglutinin
OVX: Ovariectomized
ANOVA: Analysis of variance
CHX: Cycloheximide

## References

[1] Valenti MT, Dalle Carbonare L, Mottes M (2016). Osteogenic differentiation in healthy and pathological conditions. Int J Mol Sci..

[2] Faghihi F, Baghaban EM (2014). The effect of nano-scale topography on osteogenic differentiation of mesenchymal stem cells. Biomed Pap Med Fac Univ Palacky Olomouc Czech Repub.

[3] Fu G, Ren A, Qiu Y, Zhang Y (2016). Epigenetic regulation of osteogenic differentiation of mesenchymal stem cells. Curr Stem Cell Res Ther.

[4] Martins M, Ribeiro D, Martins A, Reis RL, Neves NM (2016). Extracellular vesicles derived from osteogenically induced human bone marrow mesenchymal stem cells can modulate lineage commitment. Stem Cell Reports.

[5] Zuo R, Liu M, Wang Y, Li J, Wang W, Wu J (2019). BM-MSC-derived exosomes alleviate radiation-induced bone loss by restoring the function of recipient BM-MSCs and activating Wnt/beta-catenin signaling. Stem Cell Res Ther.

[6] Raposo G, Stoorvogel W (2013). Extracellular vesicles: exosomes, microvesicles, and friends. J Cell Biol.

[7] Liu M, Sun Y, Zhang Q (2018). Emerging role of extracellular vesicles in bone remodeling. J Dent Res.

[8] Wang X, Omar O, Vazirisani F, Thomsen P, Ekstrom K (2018). Mesenchymal stem cell-derived exosomes have altered microRNA profiles and induce osteogenic differentiation depending on the stage of differentiation. PLoS One.

[9] Finnerty JR, Wang WX, Hebert SS, Wilfred BR, Mao G, Nelson PT (2010). The miR-15/107 group of microRNA genes: evolutionary biology, cellular functions, and roles in human diseases. J Mol Biol.

[10] Gao J, Yang T, Han J, Yan K, Qiu X, Zhou Y (2011). MicroRNA expression during osteogenic differentiation of human multipotent mesenchymal stromal cells from bone marrow. J Cell Biochem.

[11] Zhi X, Chen C (2012). WWP1: a versatile ubiquitin E3 ligase in signaling and diseases. Cell Mol Life Sci.

[12] Zhao L, Huang J, Zhang H, Wang Y, Matesic LE, Takahata M (2011). Tumor necrosis factor inhibits mesenchymal stem cell differentiation into osteoblasts via the ubiquitin E3 ligase Wwp1. Stem Cells.

[13] Hou Z, Wang Z, Tao Y, Bai J, Yu B, Shen J (2019). KLF2 regulates osteoblast differentiation by targeting of Runx2. Lab Investig.

[14] Zhang X, Srinivasan SV, Lingrel JB (2004). WWP1-dependent ubiquitination and degradation of the lung Kruppel-like factor, KLF2. Biochem Biophys Res Commun.

[15] Xu R, Shen X, Si Y, Fu Y, Zhu W, Xiao T (2018). MicroRNA-31a-5p from aging BMSCs links bone formation and resorption in the aged bone marrow microenvironment. Aging Cell.

[16] Qi X, Zhang J, Yuan H, Xu Z, Li Q, Niu X (2016). Exosomes secreted by human-induced pluripotent stem cell-derived mesenchymal stem cells repair critical-sized bone defects through enhanced angiogenesis and osteogenesis in osteoporotic rats. Int J Biol Sci.

[17] Cao B, Dai X, Wang W (2019). Knockdown of TRPV4 suppresses osteoclast differentiation and osteoporosis by inhibiting autophagy through Ca^2+^-calcineurin-NFATc1 pathway. J Cell Physiol.

[18] Zhang W, Dong R, Diao S, Du J, Fan Z, Wang F (2017). Differential long noncoding RNA/mRNA expression profiling and functional network analysis during osteogenic differentiation of human bone marrow mesenchymal stem cells. Stem Cell Res Ther.

[19] Yang F, Liu DY, Guo JT, Ge N, Zhu P, Liu X (2017). Circular RNA circ-LDLRAD3 as a biomarker in diagnosis of pancreatic cancer. World J Gastroenterol.

[20] Qin Y, Wang L, Gao Z, Chen G, Zhang C (2016). Bone marrow stromal/stem cell-derived extracellular vesicles regulate osteoblast activity and differentiation in vitro and promote bone regeneration in vivo. Sci Rep.

[21] Peng S, Gao D, Gao C, Wei P, Niu M, Shuai C (2016). MicroRNAs regulate signaling pathways in osteogenic differentiation of mesenchymal stem cells (review). Mol Med Rep.

[22] Tu M, Tang J, He H, Cheng P, Chen C (2017). MiR-142-5p promotes bone repair by maintaining osteoblast activity. J Bone Miner Metab.

[23] Shu L, Zhang H, Boyce BF, Xing L (2013). Ubiquitin E3 ligase Wwp1 negatively regulates osteoblast function by inhibiting osteoblast differentiation and migration. J Bone Miner Res.

[24] Zhou Y, Liu C, He J, Dong L, Zhu H, Zhang B (2020). KLF2(+) stemness maintains human mesenchymal stem cells in bone regeneration. Stem Cells.

[25] Kim I, Kim JH, Kim K, Seong S, Kim N (2019). The IRF2BP2-KLF2 axis regulates osteoclast and osteoblast differentiation. BMB Rep.

[26] Das H, Kumar A, Lin Z, Patino WD, Hwang PM, Feinberg MW (2006). Kruppel-like factor 2 (KLF2) regulates proinflammatory activation of monocytes. Proc Natl Acad Sci U S A.

[27] Wang LM, Zhao N, Zhang J, Sun QF, Yang CZ, Yang PS (2018). Tumor necrosis factor-alpha inhibits osteogenic differentiation of pre-osteoblasts by downregulation of EphB4 signaling via activated nuclear factor-kappaB signaling pathway. J Periodontal Res.

[28] Wang YJ, Zhang HQ, Han HL, Zou YY, Gao QL, Yang GT (2017). Taxifolin enhances osteogenic differentiation of human bone marrow mesenchymal stem cells partially via NF-κB pathway. Biochem Biophys Res Commun.

[29] Engels BM, Hutvagner G (2006). Principles and effects of microRNA-mediated post-transcriptional gene regulation. Oncogene.

[30] Kang L, Yang C, Yin H, Zhao K, Liu W, Hua W (2017). MicroRNA-15b silencing inhibits IL-1beta-induced extracellular matrix degradation by targeting SMAD3 in human nucleus pulposus cells. Biotechnol Lett.

[31] Goto Y, Kojima S, Kurozumi A, Kato M, Okato A, Matsushita R (2016). Regulation of E3 ubiquitin ligase-1 (WWP1) by microRNA-452 inhibits cancer cell migration and invasion in prostate cancer. Br J Cancer.

[32] Fang SH, Chen L, Chen HH, Li YF, Luo HB, Hu DQ (2019). MiR-15b ameliorates SONFH by targeting Smad7 and inhibiting osteogenic differentiation of BMSCs. Eur Rev Med Pharmacol Sci.

[33] Vimalraj S, Partridge NC, Selvamurugan N (2014). A positive role of microRNA-15b on regulation of osteoblast differentiation. J Cell Physiol.

[34] Han Y, Zhang F, Zhang J, Shao D, Wang Y, Li S (2019). Bioactive carbon dots direct the osteogenic differentiation of human bone marrow mesenchymal stem cells. Colloids Surf B Biointerfaces.

[35] Fang S, Li Y, Chen P (2019). Osteogenic effect of bone marrow mesenchymal stem cell-derived exosomes on steroid-induced osteonecrosis of the femoral head. Drug Des Dev Ther.

